# Increased Production of Interleukin-4, Interleukin-10, and Granulocyte-Macrophage Colony-Stimulating Factor by Type 2 Diabetes' Mononuclear Cells Infected with Dengue Virus, but Not Increased Intracellular Viral Multiplication

**DOI:** 10.1155/2013/965853

**Published:** 2013-09-02

**Authors:** Ing-Kit Lee, Ching-Jung Hsieh, Rong-Fu Chen, Zih-Syuan Yang, Lin Wang, Chang-Mei Chen, Chiung-Fen Liu, Chung-Hao Huang, Chun-Yu Lin, Yen-Hsu Chen, Kuender D Yang, Jien-Wei Liu

**Affiliations:** ^1^Division of Infectious Diseases, Department of Internal Medicine, Kaohsiung Chang Gung Memorial Hospital, Kaohsiung 833, Taiwan; ^2^Chang Gung University Medical College, Tao-Yuan 333, Taiwan; ^3^Infection Control Committee, Kaohsiung Chang Gung Memorial Hospital, Kaohsiung 833, Taiwan; ^4^Division of Endocrinology & Metabolism, Department of Internal Medicine, Kaohsiung Chang Gung Memorial Hospital, Kaohsiung 833, Taiwan; ^5^Department of Medical Research, Show Chwan Memorial Hospital, Changhua 500, Taiwan; ^6^Department of Medical Research, Kaohsiung Chang Gung Memorial Hospital, Kaohsiung 833, Taiwan; ^7^Department of Pediatrics, Kaohsiung Chang Gung Memorial Hospital, Kaohsiung 833, Taiwan; ^8^Division of Infectious Diseases, Department of Internal Medicine, Kaohsiung Medical University Hospital, Kaohsiung Medical University, Kaohsiung 807, Taiwan; ^9^Graduate Institute of Medicine, College of Medicine, Kaohsiung Medical University, Kaohsiung 807, Taiwan

## Abstract

It has been reported that diabetes mellitus (DM) was an epidemiologically identified risk factor for development of dengue hemorrhagic fever (DHF)/severe dengue in dengue virus (DENV) affected patients, and T helper 2 (Th2) cytokines such as interleukin-4 (IL-4) and IL-10 each plays an important role in the immunopathogenesis of DHF in studies involving general population. To better understand the relationship between these epidemiological and immunological findings, we performed an *in vitro* study evaluating the sequential immunological reactions and viral load in the DENV infected mononuclear cells of adults with type 2 DM (T2DM group, *n* = 33) and normal adults (control group, *n* = 29). We found in the T2DM group significantly higher IL-4 level on the first (*P* = 0.049) and the third (*P* = 0.022) postinfection days, while higher IL-10 (*P* = 0.042) and granulocyte-macrophage colony-stimulating factor (GM-CSF) (*P* = 0.009) were detected on the third postinfection day. No significant difference in DENV viral load between the cultured mononuclear cells from both groups was found on the first and third post-infection days. These data immunologically suggest that patients with T2DM are at higher risk for development of DHF/severe dengue and strengthen the previously epidemiologically identified role of DM being a predictive risk factor for progressing into DHF/severe dengue in DENV-affected patients.

## 1. Introduction

Dengue is a major medical and public health problem in tropical and subtropical regions. It is estimated that approximately 50 million dengue episodes occur over the globe annually, and more than 2.5 billion people are living in geographic locales where dengue is endemic [1, 2]. There are four dengue virus serotypes (DENV-1, DENV-2, DENV-3, and DENV-4) [1, 2], and patients infected by any of the DENV serotypes may be asymptomatic or develop a wide array of clinical symptoms/signs ranging from a nonspecific febrile illness, dengue fever (DF) to dengue hemorrhagic fever (DHF). DHF is clinically characterized by bleeding and plasma leak, and a severe DHF leads to hypovolemia and even circulatory collapse in the affected patient, which is known as dengue shock syndrome (DSS) [1, 2]. Well-documented risk factors for DHF include secondary infection caused by a DENV serotype which differs from that responsible for the prior dengue episode [3, 4], the genetic predilection for causing hemorrhage of the culprit DENV [5, 6], the genetic predisposing for hemorrhage of the dengue patient [7], the aging of the host [8, 9], and diabetes mellitus (DM) [10–13]. DM is a multifaceted disease that implicates metabolic derangements and immune dysfunction [14]. The frequently found comorbidities in diabetic patients such as cardiovascular and chronic kidney diseases may add to the altered host responses to infection and clinical outcomes [15, 16]. The immunologic responses of DM patients when suffering from DENV infection have not been fully understood. It was documented that T helper (Th) cells play an important role in the immunopathogenesis of DHF [17]. Based on the types of cytokine production at activation, Th cells are divided into Th1 and Th2 [18, 19]. Activated Th1 produces IFN-*γ*, IL-2, and IL-12, whereas Th2 produces IL-4, IL-5, IL-10, and IL-13 [18, 19]. Of note, the immunologic responses in a progressive dengue patient were reported to involve a shift from the activated Th1-type cytokine response in DF to the activated Th2-type cytokine response in DHF [17, 20–24]. In general, serum levels of IFN-*γ* and IL-2 are high in patients suffering from DF, while those of IL-4, IL-6, and IL-10 remarkably upsurge in hosts experiencing severe DHF [17, 20–24]. To better understand the immune responses in dengue individuals with type 2 DM (T2DM), we investigated Th1/Th2 reactions by DENV-infected mononuclear cells of T2DM individuals. The implications of the results will be discussed.

## 2. Material and Methods

### 2.1. Ethics Statement

This study was conducted with an informed consent from all participants, which was approved by the Institutional Review Board of Chang Gung Memorial Hospital (Document no. 98-2957B).

### 2.2. Study Period and Blood Sampling

The study was conducted at Kaohsiung Chang Gung Memorial Hospital, a 2700-bed medical facility serving as a primary care and tertiary referral centre in southern Taiwan, from March through December in 2010. Participants included those with a T2DM and healthy adults, aged between 50 and 60 years. Individuals with T2DM referred to those who have been taking oral hypoglycemic agent(s) for a previously diagnosed DM [14]. Blood specimens sampled from T2DM and healthy individuals were allocated to the study group and the control group, respectively. Eight milliliters of blood were sampled from each participant. The whole blood was immediately separated into plasma and blood cells (i.e., leukocytes and erythrocytes) by centrifugation at 2,500 rpm (150 ×g) for 20 minutes. Plasma was dispensed into several aliquots and kept frozen at −80°C until being used.

### 2.3. Determination of Past DENV Infection

The serum samples of all participants were tested for dengue virus-specific immunoglobulin M (IgM) and G (IgG) antibodies using a dengue blot detection kit (Gene Labs Diagnostics, Singapore) [25, 26].

### 2.4. Separation of Mononuclear Cells

Leukocytes were separated from erythrocytes by 4.5% dextran sedimentation. After removal of erythrocytes, leukocytes were further separated into mononuclear cells and polymorphonuclear cells by density gradient centrifugation (350 g/30 min in Ficoll-Paque PLUS, Amersham Biosciences Corp.) according to standard procedures as described elsewhere [26]. Mononuclear cells were suspended in supplemented RPMI 1640 medium (Gibco BRL, Gaithersburg, MD, USA) to yield a final concentration of 1.0 × 10^6^ cells/mL for studies.

### 2.5. Preparation of DENV-2

 DENV-2 (New Guinea C strain) obtained from the Institute of Preventive Medicine, National Defense Medical Center, Taiwan, was propagated in *Aedes albopictus* C6/36 cells as previously described [27] and was used in this study. The DENV-2 viruses were harvested from the C6/36 mosquito cell-culture supernatants after incubation for 5 days. The DENV-2 titers in the supernatants were measured by a standard plaque-forming unit (pfu) assay on baby hamster kidney-21 cells. The virus titers were adjusted to a concentration of 5.0 × 10^6^ pfu/mL in RPMI 1640 medium for studies. 

### 2.6. DENV-2 Infection of Mononuclear Cells

A prior report on multiplicity of infection (MOI) of DENV ranging from 1 to 10 suggested that the higher the MOI, the simultaneously increased the DENV infection and apoptosis in the inoculated mononuclear cells [28]. To achieve a yield of sufficient DENV-infected mononuclear cells while avoiding excessive cellular apoptosis, in this experiment we used the MOI of 5, which was proven appropriate previously [29, 30]. Specifically, mononuclear cells were seeded at a density of 1.0 × 10^6^ cells/mL on 24-well plates. After an overnight incubation, the mononuclear cells were inoculated with DENV-2 from the stock with the MOI of 5 at 37°C for 2 hours [26]. The mononuclear cells were then washed twice in phosphate-buffered saline to remove cell-free viruses, and complete RPMI 1640 medium supplemented with 10% fetal bovine serum was added into each well. The infected cells were cultured in complete RPMI 1640 medium at 37°C in a 5% CO_2_ incubator. To demonstrate the innate and adaptive immunity responses *in vitro*, the supernatants and cells were harvested and analyzed on the first and third postinfection days, respectively, for measurement of responsive immune mediators and viral loads.

### 2.7. Measurement of TNF-*α*, IL-2, IL-4, IL-10, IL-12, GM-CSF, and MCP-1 Levels

In this study, the innate mediator was demonstrated by TNF-*α* [31], the Th1/Th2 reaction by IL-2, IL-4, IL-10, and IL-12 levels [19], vascular leakage mediator by MCP-1 level [32], and activated leukocytes-derived growth factor by the GM-CSF level [33]. The concentrations of TNF-*α*, IL-2, IL-4, IL-10, IL-4, GM-CSF, and MCP-l in the supernatants from the infected mononuclear cells were measured using the FlowMetrix System (Luminex Corporation, Austin, TX, USA) according to the manufacturer's instructions [34].

### 2.8. Quantitation of Viral Load by Reverse Transcription-Polymerase Chain Reaction (RT-PCR)

Viral RNA was extracted from cultured mononuclear cells to assess DENV-2 RNA viral copies by quantitative RT-PCR, as previously described [24]. The forward primer, reverse primer, and nested fluorescent probe sequences for detecting DENV-2 were 50-GGCTTAGCGCTCACATCCA-30, 50-GCTGGCCACCCTCTCTTCTT-30, and FAM-50-CGCCCACCACTATAGCTGCCGGA-30-TAMRA, respectively [24].

### 2.9. Statistical Analysis

Data are presented as mean ± SE. Student's *t*-test was used to analyze differences in immune mediators (TNF-*α*, IL-2, IL-4, IL-10, IL-4, GM-CSF, and MCP-l levels) and DENV viral load on the first and third postinfection days between the T2DM group and control groups. A *P* value of < 0.05 was considered statistically significant.

## 3. Results 

### 3.1. Demographics, Clinical, and Laboratory Information of the Participants

A total of 33 T2DM individuals (mean glycosylated hemoglobin, 7.9 ± 1.6 gm/dL) and 29 healthy individuals were recruited for this study. Participants with and without T2DM were of similar ages (mean age, 55.8 ± 2.4 years versus 54.6 ± 2.6 years; *P* = 0.083). Among the 33 T2DM participants, hypertension (63.6%) was the most common comorbidity, followed by ischemic heart disease (9.1%) and previous stroke (6.1%). All participants were negative for dengue antibody as determined by dengue blot detection kit suggesting that none of them had suffered dengue before participating in this study. 

### 3.2. Comparison of TNF-*α*, IL-2, IL-4, IL-10, IL-12, GM-CSF, and MCP-1 Levels between T2DM and Control Groups on the First and Third Postinfection Days

On the first postinfection day, no significant difference was found in concentrations of TNF-*α*, IL-2, IL-10, IL-12, GM-CSF, and MCP-l between the T2DM group and control group, but significantly higher IL-4 level (mean 1.02 ± 0.2 pg/mL versus 0.52 ± 0.13 pg/mL; *P* = 0.049) was detected in the T2DM group (Figure 1).

On the third postinfection day, the T2DM group had significantly higher IL-4 (mean 16.87 ± 4.96 pg/mL versus 4.13 ± 1.23 pg/mL; *P* = 0.022), IL-10 (mean 138.89 ± 34.62 pg/mL versus 55.49 ± 18.7 pg/mL; *P* = 0.046), and GM-CSF (mean 20.8 ± 5.3 pg/mL versus 5.1 ± 1.46 pg/mL; *P* = 0.009) levels than those of the control group. Despite nonstatistical significance, there was a trend suggesting possible higher level of vascular leakage mediator MCP-1 (mean MCP-1, 4739.75 ± 655.6 pg/mL versus 3980.8 ± 639.29 pg/mL; *P* = 0.413) in the T2DM group (Figure 2). 

### 3.3. DENV Viral Load of T2DM and Control Groups

Viral load was not detected in 1 of the specimens in T2DM group on the first and third postinfection days and in 2 and 3 specimens in the control group on the first and third postinfection days, respectively. No significant difference in detectable DENV viral load between the cultured mononuclear cells from both groups was found on the first and third postinfection days (Figure 3).

## 4. Discussion 

DM was found to be one of the many epidemiologically identified risk factors for developing severe dengue/DHF in dengue affected patients [10–13, 35]. Most of the published researches in immunology in dengue involved general population rather than a population with specific underlying disease(s) [36]. When it comes to immunopathogenesis, the role of viral burden has been controversial in DHF [21, 37, 38]. Among the multifaceted mechanism of pathogenesis of dengue, high DENV burden was reported to circumstantially associate with DHF in hosts with secondary infection [37, 38], while the overwhelming activation of Th2 cytokines was documented in the development of DHF in dengue patients of primary and secondary infections alike [17, 20–24]. Specifically, of the Th2 cytokine profile, IL-4 is the most potent cytokine in inducing Th2 cell differentiation, whereas IL-10 is responsible for anti-inflammatory reactions in the host's immune activities [21–23, 31, 36]. A significantly higher level of IL-4 found on the first postinfection day, as well as higher levels of IL-4 and IL-10 detected on the third postinfection day in the T2DM group as compared to the control group, suggests that dengue patients with an underlying T2DM are at higher risk for development of DHF, which was consistent with the same conclusion drawn based on previous epidemiological observations [10–13]. 

A number of proinflammatory cytokines/chemokines including TNF-*α*, IL-1 and IL-6, and MCP-1 were well documented to involve in the pathogenesis of diabetes mellitus [39]. GM-CSF stimulates stem cells to produce granulocytes and monocytes and plays an important role in the immune/inflammatory cascade [40]. It was reported that serum GM-CSF was significantly raised in patients with severe dengue as compared to those with mild-form dengue, and the increased GM-CSF level correlated with the development of hypotension in DHF patients [41]. The increased production of the IL-4 and the anti-inflammatory Th2-cytokine IL-10 in DENV-infected mononuclear cells of the diabetes in our study might result from a counterbalance to the comparatively highly produced pro-inflammatory cytokines/chemokines in the diabetic hosts [18, 19]. 

Limitations of this study are that the included patients were adults with a T2DM suffering from primary dengue infection, and therefore, it is uncertain whether similar immunologic responses occur in pediatric patients, in patients with type 1 DM, and/or in those with secondary dengue infection. 

In summary, this study explored the immunologic reactions in adults with T2DM experiencing primary dengue infection, and our data give insight into the immunopathogenesis of dengue in this patient population. The immunological findings suggest that patients T2DM are at higher risk for development of DHF and strengthen the previously epidemiologically identified role of DM being a predictive risk factor for progressing into DHF/severe dengue in dengue-affected patients. Stratifications of clinical severity and prediction of the risk for potential clinical deterioration are very important in a large-scale dengue epidemic happening in rural areas where medical resources are deficient, as strict observation is needed for the identified potentially risky patients so that necessary management can be delivered in a timely fashion in case of deterioration. 

## Figures and Tables

**Figure 1:** Cytokines/chemokines produced by dengue virus-infected mononuclear cells of T2DM group and control group on the first postinfection day in an *in vitro* infection model.

**Figure 2:** Cytokines/chemokines produced by dengue virus-infected mononuclear cells of T2DM group and control group on the third postinfection day in an *in vitro *infection model.

**Figure 3:** Dengue viral load in the infected mononuclear cells of T2DM group and control group on the first (a) and third (b) postinfection days in an *in vitro* infection model.
